# Investigating the Relationship between Big Five Personality Traits and Sports Performance among Disabled Athletes

**DOI:** 10.1155/2022/8072824

**Published:** 2022-05-18

**Authors:** Abdossaleh Zar, Sadeghipour Hamid Reza, Fatemeh Ahmadi, Pantelis T. Nikolaidis, Mohammad Amin Safari, Mohammad Hassan Keshazarz, Roger Ramsbottom

**Affiliations:** ^1^Department of Sport Science, School of Literature and Humanities, Persian Gulf University, Boushehr, Iran; ^2^Persian Gulf Sports, Nutrition and Health Research Core, School of Literature and Humanities, Persian Gulf University, Boushehr, Iran; ^3^School of Health and Caring Sciences, University of West Attica, Athens, Greece; ^4^Department of Sport Science, Faculty of Educational Sciences and Psychology, University of Shiraz, Shiraz, Iran; ^5^Department of Education, Federation of Veterans and Disabled, Iran; ^6^Department of Sport, Health Sciences and Social Work, Oxford Brookes University, Oxford OX3 0BP, UK

## Abstract

Awareness of the psychological issues of different groups of society can help in the management of sports programs and thus improve their athletic performance. The aim of the present study was to investigate the relationship between the big five personality traits and the sports performance of disabled athletes in team sports. Three hundred and seventy-six team athletes participated in the study. Subjects completed a questionnaire of five major personality factors, and based on the information available on the provincial boards and the Veterans and Disabled Federation, the positions obtained by each athlete were considered as a criterion for sports performance. There was a significant relationship between the flexibility factor for men and women (*r* = 0.123, *p* = 0.017), neuroticism (*r* = 0.114, *p* = 0.027), adaptation (*r* = 0.171, *p* = 0.001), extraversion (*r* = 0.157, *p* = 0.002), duty orientation (*r* = 0.104, *p* = 0.045), and sports performance at a national level. There was a significant relationship between neuroticism (*r* = 0.142, *p* = 0.006), adaptation (*r* = 0.133, *p* = 0.010), extraversion (*r* = 0.163, *p* = 0.002), and duty orientation (*r* = 0.130, *p* = 0.011) with sports performance at a provincial level. There was a significant relationship between neuroticism (*r* = 0.156, *p* = 0.002), extraversion (*r* = 0.168, *p* = 0.001), duty orientation (*r* = 0.182, *p* = 0.001), and sports performance at international level. Disabled athletes seem to have above-average performance scores in most personality factors, which can improve their physical health and increase their success in sports.

## 1. Introduction

Although psychologists acknowledge “personality” as a general concept, its definition is open to debate, with more effort being expended in actually evaluating the concept of personality [1]. Factor analysis in explaining personality structure based on traits is one of the most important and effective methods used by psychologists [2]. Researchers consider the big five main dimensions of personality to include openness to experience, neuroticism, agreeableness, extraversion, and conscientiousness. These big five factors have been shown to have good convergent validity and good separation between instrument and observer [3]. Today, this model of five major personality factors is a popular approach in the study of personality traits. In this particular model, a human is identified as a rational being who has the justification for his/her personality [4]. The model states that “man” is a rational being who can justify his/her personality and behavior [5].

In the behavioral sciences, the relationship between personality and sports behaviors of individuals has been studied as part of research conducted in the sports sciences. The five-factor personality model underlies many studies in the field of sports and personality [6]; Safari et al. [7] examined the effect of five major personality factors on the motivation of students' sports participation and reported that the five factors had a significant effect on their motivation and in total 78% of the variable changes in the motivation of students' sports participation. Shams Ravandi et al. [2] presented a structural model based on the five major personality factors to predict the “burnout” of professional football referees; they reported that personality traits with burnout through the mediation of self-esteem had a significant indirect relationship [2]. Even the relationship between personality and the choice of sports has been discussed, as it has been shown that team athletes have more factors identified with extraversion [2, 8].

Such studies show that personality factors can be very important for athletic performance. Exercise can be considered as a “laboratory” in which the performance of athletes under high pressure and with strong emotions is evaluated [9], which creates unique conditions to examine the role of personality and individual differences in athletic performance [10]. Many athletes, despite having good performance in individual or group training, have poor performance in competition, and the cause of these problems, in addition to technical problems and weakness of coaches, can be attributed to environmental and stressors affecting the mental spirit of the athlete [11]. The personality of individuals can greatly affect this athletic performance, a topic that in certain groups such as veterans and the disabled can provide an attractive field for research.

Stefanovics et al. [12] showed that the five major personality factors have a significant relationship with the body mass index (BMI) of the disabled and mentioned these factors as important factors in preventing obesity in this group. However, knowledge of the psychological issues of different groups in society can help in the management and implementation of sports programs and thus improve their athletic performance. Similarly, knowing these issues in the field of sports for the disabled and veterans can improve their athletic performance at national and international levels of competition. To date, these five personality components on the sports performance of veterans and the disabled have not been studied; therefore, the present study is aimed at investigating the relationship between the big five personality traits and the sports performance of disabled athletes in team sports.

## 2. Materials and Methods

This descriptive-analytical research (correlational study) was conducted in 2021 in Iran.

### 2.1. Participants

All disabled athletes participating in provincial, national, and international competitions made up the statistical population of the present study, of which 376 team athletes participated in the present study. Criteria for entering the study included informed consent to participate, no mental illness, and a willingness to cooperate and complete a questionnaire. All ethical considerations regarding the confidentiality of the subjects' information were observed, and the present study received ethical approval with the code IR.JUMS.REC.1399.045 from the Ethics Committee of Jahrom University of Medical Sciences (Fars Province, Iran).

### 2.2. Procedure

After the approval of the plan by the Federation of Veterans and Disabled and coordination with the sports delegations of Veterans and Disabled of the provinces, all stages of work were sent in writing to the delegations through the federation. Before data collection, the five major personality factors, as well as how to implement the research plan, were fully explained to the participants. Each volunteer completed a questionnaire of the five major personality factors [13], and based on the information available on the provincial boards and the Veterans and Disabled Federation, the positions (position refer to whether the athlete competed at provincial, national, or international level) obtained by each athlete were considered as a criterion for sports performance.

### 2.3. Questionnaire of Big Five Personality Traits

The current questionnaire identifies the big five personality traits and consists of 21 questions. The 50-item questionnaire of the five major personality factors was first developed by Goldberg [14]. And its psychometric properties in Iran were studied by Khormaee and Khayer [15] with the permission of the main creator of the questionnaire in the form of a doctoral thesis. The results of the study by Khormaee and Khayer [15] showed the high validity and reliability of this questionnaire. In addition, Khormaee and Farmani [13] based on the results of Khormaee and Khayer [15] research, by selecting the items of the questionnaire, the five major factors of Goldberg personality [14] prepared a shorter form of this questionnaire, including 25 items. The results of the factor analysis of their research confirmed the independence of the five major personality factors. The revelation of these five factors in short form is consistent with the model of the five major personality factors of Goldberg [14] and McCrae and Costa Jr [5] regarding the 50-item questionnaire. In addition, the results of factor analysis showed that four items of the short form were removed due to insufficient factor loading on the desired factor and the number of items was reduced to 21 items. In addition, the results of the reliability measure showed that the short form of the questionnaire on the five major personality factors has high reliability (from 69% for openness to experience to 83% for neuroticism and agreeableness). The five major personality factors are divided into five subscales, and the questions are measured on a 5-point Likert scale: (a) openness to experience which includes questions 5-10-14-19, (b) neuroticism which includes questions 4-9-13-18, (c) agreeableness which includes questions 2-7-16-21, (d) extraversion which includes questions 1-6-11-15-20, and (e) conscientiousness which includes questions 3-8-12-17.

### 2.4. Sports Performance

Based on the information available in the provincial sports delegations and the Veterans and Disabled Federation, the positions obtained by each athlete were considered as a criterion for sports performance.

### 2.5. Information Analysis Method

Descriptive statistics were used to determine the mean and standard deviation, and a regression correlation test (Pearson product-moment correlation coefficient) was used to investigate the relationship between research variables in the inferential statistics section. Where the data was not normally distributed, a Mann-Whitney *U* test was used to compare men versus women.

## 3. Results

### 3.1. Examination of the Five Major Personality Factors of Team Athletes

The results of the five major personality factors in women and men in team disciplines are shown in Table 1. Between openness to experience, neuroticism, agreeableness, extroversion, and conscientiousness, there was no significant difference for women compared with men.

### 3.2. Investigating the Relationship between Flexibility Factors (Related to Personality) with Sports Performance at Different Levels: Provincial, National, and International

The results showed that there was a significant relationship between the flexibility factor related to personality and athletic performance of female team athletes in the province (*r* = 0.166, *p* = 0.046), but at the national level (*r* = 0.123, *p* = 0.141) and international level (*r* = 0.041, *p* = 0.62), no significant relationship was observed (Table 2). In addition, the results showed that there was a significant relationship between personality-related flexibility to mental health, quality of life, and athletic performance of male team athletes at the national level (*r* = 0.136, *p* = 0.038), but at the provincial level (*r* = 0.045, *p* = 0.494) and international level (*r* = 0.072, *p* = 0.272), no significant relationship was observed. Also, there was a significant relationship between the flexibility factor related to personality and athletic performance of athletes (total: men and women) in team disciplines at the national level (*r* = 0.123, *p* = 0.017), but at the provincial level (*r* = 0.099, *p* = 0.055) and international level (*r* = 0.062, *p* = 0.233), no significant relationship was observed.

### 3.3. Investigating the Relationship between Neuroticism Factors (Personality Related) with Sports Performance at Different Levels: Provincial, National, and International

The results showed that between the neuroticism factor related to the personality and athletic performance of female team athletes in the province (*r* = 0.174, *p* = 0.037) and internationally (*r* = 0.215, *p* = 0.002), there was a significant relationship, but at the national level (*r* = 0.141, *p* = 0.092), no significant relationship was observed (Table 3). Between the neuroticism factor related to personality to mental health, quality of life, and athletic performance of male athletes in team disciplines in the province (*r* = 0.112, *p* = 0.087) at national (*r* = 0.091, *p* = 0.166) and international level (*r* = 0.092, *p* = 0.162), no significant relationship was observed. Moreover, between the neuroticism factor related to personality to mental health, quality of life, and sports performance of athletes (total: men and women) in team disciplines in the province (*r* = 0.142, *p* = 0.006), national (*r* = 0.114, *p* = 0.027), and international level (*r* = 0.156, *p* = 0.002), a significant relationship was observed.

### 3.4. Investigating the Relationship between Adaptation Factors (Related to Personality) with Sports Performance at Different Levels: Provincial, National, and International

There was a significant relationship between personality adjustment factor and sports performance of female team athletes at the national level (*r* = 0.267, *p* = 0.001(, but at the province (*r* = 0.30, *p* = 0.20) and international level (*r* = 0.136, *p* = 0.103), no significant relationship was observed (Table 4). The results showed that there was a significant relationship between personality adjustment factor related to mental health, quality of life, and athletic performance of male team athletes at the province level (*r* = 0.145, *p* = 0.027), but at the national (*r* = 0.094, *p* = 0.151) and international level (*r* = 0.057, *p* = 0.382), no significant relationship was observed. Furthermore, between personality adjustment factors related to mental health, quality of life, and sports performance of athletes (total: men and women) in team disciplines in the province (*r* = 0.133, *p* = 0.010) at the national level (*r* = 0.171, *p* = 0.001), there was a significant relationship, but at the international level (*r* = 0.097, *p* = 0.060), no significant relationship was observed.

### 3.5. Investigating the Relationship between Extraversion Factor (Personality Related) with Sports Performance at Different Levels: Provincial, National, and International

Between the extraversion factor related to personality and sports performance of female team athletes in the province (*r* = 0.226, *p* = 0.006) at the national (*r* = 0.358, *p* = 0.001) and international level (*r* = 0.235, *p* = 0.005), significant relationships were observed (Table 5). The results showed that between the factor of extraversion related to personality with mental health, quality of life, and athletic performance of male team athletes in the province (*r* = 0.117, *p* = 0.074) at national (*r* = 0.016, *p* = 0.814) and international level (*r* = 0.117, *p* = 0.075), no significant relationship was observed. Also, between the extroversion factor related to personality to mental health, quality of life, and sports performance of athletes (total: men and women) in team disciplines at the provincial (*r* = 0.163, *p* = 0.002), national (*r* = 0.157, *p* = 0.002), and international level (*r* = 0.168, *p* = 0.001), significant relationships were observed.

### 3.6. Investigating the Relationship between Duty-Oriented Factors (Personality Related) with Sports Performance at Different Levels: Provincial, National, and International

The results showed that between the duty-oriented factor related to personality and athletic performance of female team athletes in the province (*r* = 0.246, *p* = 0.003) at the national (*r* = 0.251, *p* = 0.002) and international level (*r* = 0.138, *p* = 0.001), significant relationships were observed (Table 6). The results showed that between the duty-oriented factor related to personality to mental health, quality of life, and athletic performance of male team athletes in the province (*r* = 0.044, *p* = 0.502) at the national level (*r* = 0.00, *p* = 0.998), no significant relationship was observed, but at the international level (*r* = 0.211, *p* = 0.001), a significant relationship was observed (Table 6). The results showed that between the factor of duty orientation related to personality and sports performance of athletes (total: men and women) in team disciplines in the province (*r* = 0.30, *p* = 0.011) at the national (*r* = 0.104, *p* = 0.045) and international level (*r* = 0.182, *p* = 0.001), significant relationships were observed (Table 6).

## 4. Discussion

In the present study, the relationship between the big five major personality factors and sports performance of veterans and athletes with a disability was investigated. The results of the present study showed a significant relationship between the openness and athletic performance of the athlete's team (total: men and women) at the national level. But there was a significant difference between the three factors of neuroticism, extraversion, and conscientiousness with the sports performance of athletes (total: men and women) in all three levels of competition, and there was a significant relationship in the factor of agreeableness at both province and national level.

In a research by Safari et al. [7], it was shown that these five factors have a significant effect on the motivation of students' sports participation. In the study of Keshavarz et al. [16], there was a significant difference in neuroticism of Iranian and non-Iranian athletes, but there was no significant difference in this characteristic in Iranian student-athletes. According to McCrae and Costa [3], people who score higher on neuroticism are anxious, timid, and prone to panic and anxiety. They also cannot cope well with everyday stress, helplessness, and embarrassment. According to the findings of the present study, it seems that elite veteran male and female athletes are of “high quality,” which can pave the way for their success.

Fazel [1] compared these five major personality factors between male and female athletes and reported that, except for the personality factor of openness, there was a significant difference between athletes and nonathletes in four other factors. Jackson et al. [17] also showed that there was a significant difference between the personality factor of openness in athlete and nonathlete groups. However, these findings are inconsistent with the results of Kajtna et al. [18] and Reiter et al. [19]. Nevertheless, the nature of sports and physical activity seems to satisfy people's inner emotions through more openness, an increase in the desire for more experiences and learned techniques, and increased motivation to participate in social arenas such as sports that this issue in veteran and disabled athletes can have a positive effect on their athletic performance.

In the study of Lewis and Sutton [20] and also Ghaderi and Ghaderi [6] in line with the present study, it was shown that personality factors such as extraversion are higher in athletes, and it links with greater sports participation. Extroverts gain extra energy from connecting with the outside world and exposing themselves to social activities. Therefore, it seems that veterans and the disabled, due to having a higher score in this personality trait, have good sports performance and can achieve high levels at the national and international levels in the field of sports. Brinkman [21] also reported a significantly higher conscientiousness personality factor in athletes. Conscientious people have a great desire to control their emotions and focus on their goals and thus have a higher sense of responsibility and try to perform in the best possible way in their assigned tasks [7]. It seems that the highest score of this personality trait in veterans and athletes with disabilities can have a positive effect on their performance and help them to be more successful in the field of sport. Agreeableness was also mentioned in line with this research by Ghaderi and Ghaderi [6] as a personality trait that affects athletic performance. Agreeableness shows the level of cooperation and friendly attitude, and people with higher agreeableness have a high tendency to participate in team sports, which can have a positive effect on their performance. This finding was also shown in the present study of veteran and disabled athletes.

As mentioned, this questionnaire examined the five major personality factors (openness to experience, neuroticism, agreeableness, extraversion, and conscientiousness) among disabled athletes. It seems that the high score obtained in this questionnaire for some factors, such as openness to experience, reflects disabled athletes' physical and motivational limitations, which in turn may cause them frustration within society. These findings highlight the need to help these people to show their innate ability by experiencing new sports environments and gain the respect and admiration of people in the community. In addition, it has been observed that, in general, the factor of extraversion is higher in athletes than nonathletes, and disabled athletes are more inclined to participate in sports activities [1, 17–19]. Therefore, it seems that disabled athletes with a higher score in this factor have a high motivation to participate in sports activities and be able to achieve high success by participating in national and international competitions. In addition, people with disabilities have a high sense of duty and try to be able to best fulfill the responsibilities assigned to them, and this feature can have a significant impact on the national and international success of these athletes [7]. In people with disabilities, due to their disabilities, the spirit of cooperation is very high, so these people have a high score in agreement, and this high score affects their success in national and international competitions [6].

Based on the findings of the present study, it seems that disabled athletes have above-average performance scores in most personality factors, which indicates that sport and physical activity in this group of society can not only improve their level of physical and mental health but also increase their success in domestic and international sports participation. This finding should be given special attention in the planning of a country's sports officials and plans for the competition.

## Figures and Tables

**Table 1:** Examining the five major personality factors (mean ± standard deviation) in team athletes.

Variable	Women	Men	Women+men	*p*
Openness to experience	12.51 ± 3.02	12.66 ± 1.96	12.60 ± 2.42	0.618
Neuroticism	12.85 ± 2.52	12.88 ± 2.00	12.87 ± 2.226	0.899
Agreeableness	12.31 ± 2.05	12.34 ± 1.35	12.33 ± 1.65	0.839
Extraversion	18.08 ± 3.20	18.22 ± 2.72	18.16 ± 2.91	0.681
Conscientiousness	12.72 ± 2.40	12.40 ± 2.14	12.52 ± 2.25	0.185

**Table 2:** Investigating the relationship between flexibility factor and sports performance at different levels: provincial, national, and international.

Variable	Group	Sports performance at the provincial level		Sports performance at the national level		Sports performance at the international level	
		*r*	*p*	*r*	*p*	*r*	*p*
Flexibility	Women	0.166	0.046^∗^	0.123	0.141	0.041	0.628
	Men	0.045	0.494	0.136	0.038^∗^	0.072	0.22
	Women+men	0.099	0.055	0.123	0.017^∗^	0.062	0.232

^∗^Indicates a significant relationship between the two variables.

**Table 3:** Investigating the relationship between neuroticism factors and sports performance at different levels: provincial, national, and international.

Variable	Group	Sports performance at the provincial level		Sports performance at the national level		Sports performance internationally	
		*r*	*p*	*r*	*p*	*r*	*p*
Neuroticism	Women	0.174	0.037^∗^	0.141	0.092	0.251	0.002^∗^
	Men	0.112	0.087	0.091	0.166	0.092	0.162
	Women+men	0.142	0.006^∗^	0.114	0.027^∗^	0.156	0.002^∗^

^∗^Indicates a significant relationship between the two variables.

**Table 4:** Investigating the relationship between adaptation factors and sports performance at different levels: provincial, national, and international.

Variable	Group	Sports performance at the provincial level		Sports performance at the national level		Sports performance at the international level	
		*r*	*p*	*r*	*p*	*r*	*p*
Adaptation	Women	0.130	0.120	0.267	0.001^∗^	0.136	0.130
	Men	0.145	0.027^∗^	0.094	0.151	0.057	0.382
	Women+men	0.133	0.010^∗^	0.171	0.001^∗^	0.097	0.060

^∗^Indicates a significant relationship between the two variables.

**Table 5:** Investigating the relationship between extraversion factor and sports performance at different levels: provincial, national, and international.

Variable	Group	Sports performance at the provincial level		Sports performance at the national level		Sports performance at the international level	
		*r*	*p*	*r*	*p*	*r*	*p*
Extraversion	Women	0.226	0.006^∗^	0.385	0.001^∗^	0.235	0.005^∗^
	Men	0.117	0.074	0.016	0.814	0.117	0.075
	Women+men	0.163	0.002^∗^	0.157	0.002^∗^	0.168	0.001^∗^

^∗^Indicates a significant relationship between the two variables.

**Table 6:** Investigating the relationship between the duty-oriented factor and sports performance at levels: provincial, national, and international.

Variable	Group	Sports performance at the provincial level		Sports performance at the national level		Sports performance at the international level	
		*r*	*p*	*r*	*p*	*r*	*p*
Duty-oriented	Women	0.246	0.003^∗^	0.251	0.002^∗^	0.138	0.001^∗^
	Men	0.044	0.502	0.000	0.998	0.211	0.001^∗^
	Women+men	0.130	0.011^∗^	0.104	0.045^∗^	0.182	0.001^∗^

^∗^Indicates a significant relationship between the two variables.

## Data Availability

Data will be available from the corresponding author if required.
